The article "Baricitinib protects mice from sepsis-induced cardiac dysfunction and multiple-organ failure" was retracted in 2024. Reasons: duplicated images; unreliable data; unreliable results or conclusions; concerns about the images.

# Baricitinib protects mice from sepsis-induced cardiac dysfunction and multiple-organ failure

**DOI:** 10.3389/fimmu.2023.1223014

**Published:** 2023-09-12

**Authors:** Chiara Verra, Shireen Mohammad, Gustavo Ferreira Alves, Elisa Porchietto, Sina Maren Coldewey, Massimo Collino, Christoph Thiemermann

**Affiliations:** ^1^ William Harvey Research Institute, Barts and The London School of Medicine and Dentistry, Queen Mary University of London, London, United Kingdom; ^2^ Department of Neurosciences “Rita Levi Montalcini”, University of Turin, Turin, Italy; ^3^ Pharmacology Unit, School of Pharmacy, University of Camerino, Camerino, Italy; ^4^ Department of Anesthesiology and Intensive Care Medicine, Jena University Hospital, Jena, Germany; ^5^ Septomics Research Center, Jena University Hospital, Jena, Germany

**Keywords:** sepsis, baricitinib, Janus Kinase, cardiac dysfunction, multiple-organ failure

## Abstract

Sepsis is one of the major complications of surgery resulting in high morbidity and mortality, but there are no specific therapies for sepsis-induced organ dysfunction. Data obtained under Gene Expression Omnibus accession GSE131761 were re-analyzed and showed an increased gene expression of Janus Kinase 2 (JAK2) and Signal Transducer and Activator of Transcription 3 (STAT3) in the whole blood of post-operative septic patients. Based on these results, we hypothesized that JAK/STAT activation may contribute to the pathophysiology of septic shock and, hence, investigated the effects of baricitinib (JAK1/JAK2 inhibitor) on sepsis-induced cardiac dysfunction and multiple-organ failure (MOF). In a mouse model of post-trauma sepsis induced by midline laparotomy and cecal ligation and puncture (CLP), 10-week-old male (n=32) and female (n=32) C57BL/6 mice received baricitinib (1mg/kg; i.p.) or vehicle at 1h or 3h post-surgery. Cardiac function was assessed at 24h post-CLP by echocardiography *in vivo*, and the degree of MOF was analyzed by determination of biomarkers in the serum. The potential mechanism underlying both the cardiac dysfunction and the effect of baricitinib was analyzed by western blot analysis in the heart. Trauma and subsequent sepsis significantly depressed the cardiac function and induced multiple-organ failure, associated with an increase in the activation of JAK2/STAT3, NLRP3 inflammasome and NF- κβ pathways in the heart of both male and female animals. These pathways were inhibited by the administration of baricitinib post the onset of sepsis. Moreover, treatment with baricitinib at 1h or 3h post-CLP protected mice from sepsis-induced cardiac injury and multiple-organ failure. Thus, baricitinib may be repurposed for trauma-associated sepsis.

The article "Baricitinib protects mice from sepsis-induced cardiac dysfunction and multiple-organ failure" was retracted in 2024. Reasons: duplicated images; unreliable data; unreliable results or conclusions; concerns about the images.

## Introduction

Sepsis is defined as a life-threatening organ dysfunction caused by an infection leading to activation of the host’s immune system with an excessive inflammatory response (cytokine storm) often followed by immune paralysis (1–3). Every year, 50 million cases of sepsis occur worldwide resulting in 11 million deaths (4). Sepsis is one of the most common complications after trauma leading to increased morbidity and mortality (5–9). Approximately 50% of septic patients exhibit signs of cardiac dysfunction, with ventricular dilation, reduced contractility and diastolic dysfunction, which are associated with an increased mortality (10–12). Most notably, sepsis-related cardiac dysfunction drives tissue hypoperfusion and multi-organ damage (13–15). The pathogenesis of the myocardial dysfunction in sepsis is not entirely clear, as it is associated with molecular and metabolic alterations as well as microcirculatory changes (16, 17). However, one of the main cause of sepsis-driven myocardial dysfunction is the cytokine storm, that directly depresses myocardial contractility (18–20). Indeed, sepsis mainly differs from a local infection by an uncontrolled and excessive immune response, characterized by massive release of pro-inflammatory cytokines (e.g. IL-1β and TNFα), which drives excessive systemic inflammation, which can lead to multiple organ failure (MOF) and death (21).

In 2019, an enormous threat to global health spread worldwide, namely COVID-19 (driven by the virus SARS-CoV-2) (22). This new systemic viral infection can also trigger a cytokine storm leading to sepsis and resulting in MOF and death (23). For this reason, management of cytokine release syndrome caused by SARS-CoV-2 infection has been explored as a potential treatment of COVID-19 (24). With this in mind, the efficacy of a number of anti-inflammatory interventions (repurposing) has been evaluated in patients with COVID-19 (25–27). In particular, baricitinib, an inhibitor of Janus Kinase (JAK)1 and JAK2 and licensed in many countries for the treatment of rheumatoid arthritis, atopic dermatitis and alopecia areata, has been reported to reduce the mortality in COVID-19 patients (28–31). Indeed, the JAK family, composed of JAK1, JAK2, JAK3 and tyrosine kinase 2 (TYK2), is involved, together with the signal transducer and activator of transcription (STAT), in the intracellular signaling cascade triggered by circulating pro-inflammatory mediators associated with the cytokines storm induced by SARS-CoV-2 (32).

We have recently reported that JAK/STAT inhibition by baricitinib reduces the post-traumatic multiple-organ dysfunction in a rat model of hemorrhagic shock (33). We report here for the first time that post-operative patients that developed sepsis exhibit an increase in the expression of elements of the JAK-STAT pathway. Thus, we hypothesized that JAK/STAT activation may contribute to the pathophysiology of septic shock and, given the lack of specific therapies for sepsis-induced MOF, that baricitinib may be a potential treatment (34). We have subsequently used a clinically relevant, murine sepsis model to investigate the effects of baricitinib on cardiac dysfunction and multiple-organ failure. Moreover, we examined the possible molecular mechanism of action of the observed effects of baricitinib by analyzing the activation of both NF-kB and NLRP3 inflammasome in our murine model of sepsis. Finally, we also evaluated the potential gender differences in responses to sepsis and therapeutic intervention in these mice.

The article "Baricitinib protects mice from sepsis-induced cardiac dysfunction and multiple-organ failure" was retracted in 2024. Reasons: duplicated images; unreliable data; unreliable results or conclusions; concerns about the images.

## Materials and methods

### JAK2 and STAT3 gene expression in human whole blood of septic shock patients

Original data were obtained under Gene Expression Omnibus (GEO) accession GSE131761, published by Martínez-Paz et al. (35). Whole blood was collected from post-operative patients (n=81) 24h after diagnosis of septic shock and from healthy volunteers (n=15). Total RNA was extracted from blood samples and hybridized with Agilent Whole Human Genome Oligo Microarray Kit following manufacturer’s instructions. JAK1/2 and STAT3 gene expression data were analyzed to compare the results between septic patients and healthy volunteers.

### Animals and ethical statement

This study included equal numbers of 10-week-old male (n=32) and female (n=32) C57BL/6 mice (Charles River, UK), weighing 20-30g, kept under standard laboratory conditions as previously described (36). The Animal Welfare Ethics Review Board of Queen Mary University of London (QMUL) approved all the *in vivo* experiments in accordance with the Home Office guidance on the Operation of Animals (Scientific Procedures Act 1986) published by Her Majesty’s Stationery Office and the Guide for the Care and Use of Laboratory Animals of the National Research Council. All research was conducted under U.K. Home Office project license number PP6747232. All *in vivo* experiments are reported in accordance to ARRIVE guidelines (37).

### Cecal ligation and puncture surgery

Cecal Ligation Puncture (CLP) is a surgical procedure used in rodents for reproducing the clinical course of sepsis (38). After injection of buprenorphine, anesthesia was induced (inhalation of 3% isoflurane) and maintained with isoflurane [2% and oxygen (1L/min)]. Fur was removed and the abdomen of the animals was opened (1.5cm midline incision), the cecum was ligated below the ileo-cecal valve, perforated at the top and at the bottom (18G needle) and gently squeezed to extrude a small amount of feces from both sides. Then, the caecum was returned to the peritoneal cavity in its anatomical position and 5mL/kg of pre-warmed saline was administered into the abdomen before closure. After surgery, pre-warmed normal saline (10mL/kg; s.c.) was administered as fluid resuscitation.

The article "Baricitinib protects mice from sepsis-induced cardiac dysfunction and multiple-organ failure" was retracted in 2024. Reasons: duplicated images; unreliable data; unreliable results or conclusions; concerns about the images.

### Experimental design

Mice were randomly divided into 4 groups of 16 animals each, containing equal number of male (n=8) and female (n=8) animals: Sham+vehicle (5% DMSO + 95% normal saline; i.p), CLP+vehicle (5% DMSO + 95% normal saline; i.p), CLP+1hBar and CLP+3hBar (1 mg/kg baricitinib dissolved in 5% DMSO + 95% normal saline; i.p.; administered at 1h or 3h after CLP). Temperature and body weight were measured, and buprenorphine (0.05mg/kg, i.p.) was given as analgesic. Sham+vehicle animals were subjected to laparotomy without CLP. Antibiotics (imipenem/cilastatin; 2mg/kg dissolved in resuscitation fluid saline) and the analgesic (buprenorphine) were injected via s.c. and i.p. respectively, 6h and 18h after CLP or sham surgery. Just before echocardiography, sepsis severity was evaluated using the murine sepsis score (MSS) (39). A MSS of < 1 indicates a mild condition, a score between 1 and 3 denotes moderate sepsis, and a MSS of ≥ 3 indicates severe sepsis. Cardiac function was then assessed (see below). After echocardiography, mice were deeply sedated prior to cardiac puncture to obtain blood samples. Mice were then killed by removal of heart and lungs, and the heart was collected to be stored at low temperature (-80°C) for further analysis (**Figure 2A**).

### Assessment of cardiac function *in vivo* and quantification of multiple-organ injury/dysfunction

Echocardiography was performed *in vivo* at 24h after CLP, by using the Vevo-3100 imaging system and MX550D transducer (FujiFilm Visualsonics), as previously described (36). Cardiac function was analyzed by measuring ejection fraction (EF%), fractional shortening (FS%), cardiac output (CO) and stroke volume (SV) of the left ventricle. At the end of the echocardiography, serum samples were obtained to assess the multiple-organ injury and dysfunction in all mice as previously described (40, 41), by an independent veterinary testing laboratory (MRC (Medical Research Council) Harwell Institute, Oxford, England) to quantify creatinine, alanine aminotransferase (ALT) and aspartate aminotransferase (AST), creatine kinase (CK) and lactate dehydrogenase (LDH).

### Western blot analysis

Total, cytosolic and nuclear extractions from heart tissue were quantified by BCA protein assay, following the manufacturer’s instructions (23225 Pierce^®^ BCA Protein, Pierce Biotechnology Inc., Rockford, IL, USA). As previously described (42), equal amounts of proteins (50µg) were separated by sodium dodecyl sulphate polyacrylamide gels (SDS-PAGE) at the percentages of either 8% or 10% and transferred by polyvinylidene difluoride membranes (GE10600038 Amersham™ Hybond^®^ P Western blotting membranes, PVDF; Merck, Darmstadt, Germany). Membranes were blocked for 1h and incubated (overnight) with the primary antibodies (see **Supplementary Material**; **Supplementary Table 1**). Blots were incubated with HRP conjugated secondary antibody (anti-rabbit #7074, anti-mouse #7076). Chemiluminescence signal was detected by using ECL system (Bio-Rad Laboratories, Inc., Hercules, CA 94547, USA) and bands were quantified through ImageLab Version 6.1.0 BioRad Laboratories Software. Results were normalized to respective housekeepings.

The article "Baricitinib protects mice from sepsis-induced cardiac dysfunction and multiple-organ failure" was retracted in 2024. Reasons: duplicated images; unreliable data; unreliable results or conclusions; concerns about the images.

### Statistical analysis

All data in text and figures were expressed as mean ± standard error mean (SEM) of n observations, where n represents the number of patients/animals. All the statistical analyses were made on GraphPad Prism 9 (GraphPad Software, Inc., La Jolla, CA, USA). Statistical differences were analyzed by unpaired *t*-test or using one-way ANOVA followed by a Bonferroni’s *post-hoc* test, as appropriate. Pearson’s correlation with *P*-values based on two tailed test was used to determine correlations coefficients. None of the animals died and no data were excluded from the study. All values with a P-value less than 0.05 were considered statistically significant.

## Results

### JAK2 and STAT3 gene expression increases in post-operative septic shock patients

Martínez-Paz et al. collected whole blood of post-operative patients with confirmed septic shock and of healthy volunteers to evaluate gene expression patterns (35). We reanalyzed the dataset for JAK1, JAK2 and STAT3 expression and found that, when compared to healthy volunteers, JAK1 gene expression was not significantly increased in post-operative patients with confirmed septic shock (data not shown). In contrast, the expression of JAK2 and STAT3 (downstream of JAK2 and stimulated by activation of JAK2) were significantly increased in patients with septic shock when compared to healthy volunteers in both genders (P<0.0001; **Figures 1A–D**). These results point to a potential role of the JAK2-STAT3 pathway in the pathophysiology of septic shock.

**Figure 1:** JAK2 and STAT3 gene expression is elevated in post-operative septic shock patients. Data were taken from the Gene Expression Omnibus under dataset accession number GSE131761, published by Martínez-Paz and colleagues. RNA was extracted from whole blood of (total n=81 patients, of which n=48 male and n=33 female patients) post-operative septic shock patients (Septic Shock group) and from (total n=15, of which n=10 male and n=5 female healthy volunteers) healthy volunteers (Healthy group) of mixed age. **(A, B)** Differences in JAK2 **(A)** and STAT3 **(B)** gene expression between healthy volunteers and post-operative septic shock patients of both genders. **(C, D)** Differences in JAK2 **(C)** and STAT3 **(D)** gene expression between male healthy volunteers and post-operative septic shock patients and female healthy volunteers and post-operative septic shock patients. Statistical differences between the groups (Healthy and Septic Shock) were analyzed by unpaired t-test or using one-way ANOVA followed by a Bonferroni’s *post-hoc* test, as appropriate. A value of ****P<0.0001 was statistically significant.

The article "Baricitinib protects mice from sepsis-induced cardiac dysfunction and multiple-organ failure" was retracted in 2024. Reasons: duplicated images; unreliable data; unreliable results or conclusions; concerns about the images.

### Baricitinib reduces sepsis-induced cardiac dysfunction when administered either 1h or 3h post-CLP

The ability of the left ventricle to pump enough blood out through the aorta was assessed by echocardiography *in vivo* 24h after CLP or sham surgery (**Figure 2A**). The EF%, FS%, CO and SV were measured by analyzing the M-mode traces obtained (**Figure 2B**), which showed the differences in the systolic contraction of the left ventricle in the four groups considered. When compared to sham-operated mice, mice subjected to CLP and treated with vehicle (CLP+vehicle) demonstrated a significant reduction in EF%, FS%, CO and SV (P<0.0001; **Figures 2C–F**), indicating the development of systolic, cardiac dysfunction. In contrast, treatments of CLP-mice with baricitinib either 1h or 3h post-surgery significantly reduced the decline in all these cardiac parameters (P<0.0001; **Figures 2C–F**) caused by CLP and detected in CLP+vehicle mice. The decline in EF% was associated with an increase in MSS and a fall in body temperature measured at 24h after CLP (**Figures 2G–J**).

**Figure 2:** Baricitinib reduces sepsis-induced cardiac dysfunction when administered 1h or 3h post-CLP. Mice were treated with vehicle or baricitinib (1mg/kg; i.p.) either 1h or 3h after CLP. **(A)** Experimental design. **(B)** Schematic representations of the left ventricle taken in M-mode of the four groups. **(C–H)** The graphs display the differences between the groups in terms of ejection fraction (%), fractional shortening (%), cardiac output, stroke volume, body temperature at 24h and murine sepsis score (MSS). The following groups containing equal number of male and female mice were studied: sham+vehicle (n=16), CLP+vehicle (n=16), CLP+1hBaricitinib (n=16) and CLP+3hBaricitinib (n=16). A value of ****P<0.0001 was statistically significant when compared to CLP+vehicle by one-way ANOVA followed by a Bonferroni’s post hoc test. **(I)** Correlation between MSS and EF%, **(J)** correlation between temperature at 24h and EF%. Correlations coefficients were determined by Pearson’s correlation with P-value based on two-tailed tests.

The article "Baricitinib protects mice from sepsis-induced cardiac dysfunction and multiple-organ failure" was retracted in 2024. Reasons: duplicated images; unreliable data; unreliable results or conclusions; concerns about the images.

### Baricitinib attenuates hepatocellular injury and protects mice from renal dysfunction when administered 1h or 3h after CLP

Biomarkers of hepatocellular injury (ALT and AST), renal dysfunction (creatinine), skeletal muscle injury (CK) and cell-death (LDH) were analyzed in the serum. When compared to sham-operated mice, mice subjected to CLP and treated with vehicle developed kidney dysfunction, hepatocellular injury, skeletal muscle injury and cellular damage (P<0.0001; **Figures 3A–E**). When compared to CLP+vehicle, treatment of CLP-mice with baricitinib at 1h after onset of sepsis significantly reduced the organ dysfunction/injury caused by sepsis (P<0.0001; **Figures 3A–E**). Administration of baricitinib as late as 3h after CLP also reduced the organ injury/dysfunction caused by sepsis, although the effect was less pronounced (P<0.0001; **Figures 3A–E**).

**Figure 3:** Baricitinib attenuates sepsis-induced multi-organ dysfunction. Mice were treated with vehicle or Baricitinib (1mg/kg; i.p.) either 1h or 3h after. 24h after CLP, blood samples were collected to evaluate the amount of **(A)** aspartate transaminase (AST), **(B)** alanine aminotransferase (ALT), **(C)** creatinine, **(D)** creatine kinase (CK) and **E**) lactate dehydrogenase (LDH). The following groups containing equal number of male and female mice were studied: sham+vehicle (n = 16), CLP+vehicle (n = 16), CLP+1hBaricitinib (n=16) and CLP+3hBaricitinib (n=16). All data are expressed as mean ± SEM for n number of observations. A value of ****P<0.0001 was statistically significant when compared to CLP+vehicle by one-way ANOVA followed by a Bonferroni’s post hoc test.

### Baricitinib reduces JAK/STAT pathway activation in the heart of both genders CLP animals

Clinical data showed that JAK2 and STAT3 are upregulated in septic patients. Moreover, we reported here that baricitinib protects mice from sepsis-induced cardiac dysfunction. Thus, we investigated (by western blot analysis) whether CLP leads to activation of the JAK2/STAT3 pathway in the heart. When compared to sham-operated mice, phosphorylation of JAK2 at Tyr^1007/1008^ and STAT3 at Tyr^705^ was significantly increased in the hearts of male and female mice subjected to sepsis (CLP+vehicle; P<0.001; **Figures 4A, B**). Baricitinib given 1h post-CLP significantly decreased the phosphorylation of these proteins in the heart of both genders in a similar manner (P<0.001; **Figures 4A, B**).

The article "Baricitinib protects mice from sepsis-induced cardiac dysfunction and multiple-organ failure" was retracted in 2024. Reasons: duplicated images; unreliable data; unreliable results or conclusions; concerns about the images.

**Figure 4:** Baricitinib reduces JAK/STAT and abolishes NF-κB and NLRP3 activation in both genders CLP-animals. Mice were treated with vehicle or baricitinib (1mg/kg; i.p.) 1h after CLP. Western blot analyses were conducted on cardiac tissue of animals of both genders to determine **(A)** phosphorylation of JAK2 at Tyr^1007-1008^; **(B)** phosphorylation of STAT3 at Tyr^705^; **(C)** expression of NLRP3; **(D)** activation of caspase-1; **(E)** phosphorylation of IκBα at Ser32/36; **(F)** nuclear translocation of p65. Protein expression was measured as relative optical density (O.D.) and normalized to the sham band. The following groups of male and female animals were studied: sham+vehicle (n=4), CLP+vehicle (n=5) and CLP+1hBaricitinib (n=5). All data are expressed as mean ± SEM for n number of observations. A value of ****P<0.0001, *** P<0.001, **P<0.01 was statistically significant when compared to CLP+vehicle by one-way ANOVA followed by a Bonferroni’s post hoc test.

### Baricitinib abolishes the activation of cardiac key signaling inflammatory pathways in male and female CLP-animals

The effect of JAK/STAT inhibition on the cardiac activation of NF-ĸB and NLRP3 inflammasome, two key inflammatory pathways activated in sepsis, was assessed. When compared to sham-operated mice, NLRP3 inflammasome expression and cleaved caspase-1 significantly increased in CLP+vehicle animals of both genders (**P<0.01; **Figures 4C, D**). Moreover, vehicle treated male and female CLP-animals showed increased phosphorylation of IκBα at Ser^32/36^ and translocation of p65 to the nucleus compared to sham-animals (**P<0.01; **Figures 4E, F**). When compared to CLP+vehicle animals, baricitinib treatment 1h post-CLP significantly inhibited these increases in both genders (**P<0.01; **Figures 4C–F**).

### The degree of protection afforded by baricitinib is similar in both genders

Male and female mice were used to evaluate any potential gender differences in either a) degree of organ dysfunction/injury, or b) treatment response. CLP induced a similar degree of cardiac-dysfunction, renal dysfunction and liver injury in both male and female mice when compared to sham-operated mice of the related gender (P<0.0001; **Figures 5A–D**). Moreover, the degree of reduction in organ dysfunction afforded by baricitinib (when given either 1h or 3h after the onset of sepsis) was similar in male and female CLP-animals (P<0.05; **Figures 5A–D**).

**Figure 5:** Baricitinib protects mice from CLP-induced sepsis in both genders. Mice were treated with vehicle or baricitinib (1mg/kg; i.p.) either 1h or 3h after CLP. **(A–D)** The graphs display the differences between the groups devided by genders in terms of Ejection Fraction % (EF%), alanine aminotransferase (ALT), creatinine and lactate dehydrogenase (LDH). The following groups of male and female animals were studied: sham+vehicle (n=8), CLP+vehicle (n = 8), CLP+1hBaricitinib (n = 8) and CLP+3hBaricitinib (n = 8). All data are expressed as mean ± SEM for n number of observations A value of ****P<0.0001, *** P<0.001, **P<0.01, *P<0.05 was statistically significant when compared to the CLP+vehicle by one-way ANOVA followed by a Bonferroni’s post hoc test.

The article "Baricitinib protects mice from sepsis-induced cardiac dysfunction and multiple-organ failure" was retracted in 2024. Reasons: duplicated images; unreliable data; unreliable results or conclusions; concerns about the images.

## Discussion

We have used the GEO database to gain a better understanding of any potential alterations in the expression of key elements of the JAK/STAT pathway in whole blood in healthy volunteers or in patients with sepsis after surgery. We report here for the first time, that patients with post-operative sepsis have an enhanced expression of JAK2 and STAT3 (**Figure 1**). Moreover, we have recently reported that JAK2 and STAT3 are highly expressed in trauma patients with complicated recovery, and that the JAK1/2 inhibitor baricitinib ameliorates the organ injury/dysfunction associated with hemorrhagic shock in a well-established rat model (33, 43, 44). Based on the above, we hypothesized that activation JAK/STAT may contribute to the pathophysiology of septic shock and, hence, investigated the effects of baricitinib on cardiac dysfunction and multiple-organ failure (MOF) in a surgical, murine model of sepsis. The model comprises of a surgical event (laparotomy and CLP) followed by infection in order to recreate a clinically relevant murine model of post-operative sepsis with fluid resuscitation, antibiotics and analgesics.

We report here for the first time that baricitinib reduces the CLP-induced cardiac dysfunction, measured as decline in EF%, FS%, CO and SV (**Figures 2C–F**), either when administered as an early treatment (1h post-surgery) or as a late intervention (at 3h after the onset of sepsis). Furthermore, the decline in EF% was associated with an increase in the severity of illness (MSS) and a fall in body temperature measured at 24h after CLP **(Figures 2I, J**). When administered 1h post-CLP, baricitinib abolished sepsis-induced hypothermia and MSS (**Figures 2G, H**). In addition to preventing the development of cardiac dysfunction in sepsis, baricitinib (1h or 3h after CLP) also attenuated renal dysfunction, hepatocellular injury, skeletal muscle injury (**Figures 3A–E**) associated with sepsis. The development of organ injury and dysfunction also positively correlated with the increase in MSS and negatively correlated with the fall in body temperature (see **Supplementary Material**; **Supplementary Figures 1**, **2**).

The article "Baricitinib protects mice from sepsis-induced cardiac dysfunction and multiple-organ failure" was retracted in 2024. Reasons: duplicated images; unreliable data; unreliable results or conclusions; concerns about the images.

Having discovered that baricitinib reduces MOF in sepsis, we investigated the mechanisms underlying the observed therapeutic effect. The JAK1/JAK2 inhibitor, baricitinib, was designed to treat inflammatory diseases and is currently licensed for the treatment of rheumatoid arthritis, severe atopic dermatitis, severe alopecia areata (45–49) and recently received emergency FDA approval for COVID-19 (50). Therefore, we investigated the impact of sepsis and/or baricitinib on the activation of the JAK/STAT pathway (the target for the drug) and on further inflammatory pathways known to play a crucial role in the pathophysiology of sepsis-induced cardiac (and multi-organ) dysfunction, namely NF-κB and NLRP3 inflammasome. CLP-induced sepsis resulted in a significant increase in cardiac JAK2/STAT3 activity (measured as increase in phosphorylation at Tyr^1007/1008^ for JAK2 and at Tyr^705^ for STAT3), which was reduced by baricitinib (**Figures 4A, B**). Inhibition of JAK2/STAT3 activity with baricitinib was associated with reduced activation of NF-κB and assembly and activation (caspase-1 formation) of the NLRP3 inflammasome in the heart of CLP-animals (**Figures 4C–F**).

These findings not only demonstrate the drug ability of the pharmacological target in our experimental conditions but also confirm the relevant crosstalk mechanisms linking JAK2/STAT3 activity to the modulation of other sepsis-related inflammatory cascades. Indeed, there is good evidence of interplay between JAK2/STAT3 and NF-κB pathways in inflammatory diseases (51, 52). Specifically, STAT3 has been demonstrated to be involved in the acetylation of the p65 NF-κB subunit in the nucleus, hence allowing persistent NF-kB nuclear activity (53), resulting in the expression of pro-inflammatory mediators, which may significantly contribute to systemic inflammation and organ injury-dysfunction in sepsis (54–56). We report here that both the phosphorylation of IκBα at Ser^32/36^ and the increase in the nuclear translocation of p65 in the cardiac tissue caused by sepsis were diminished by baricitinib (**Figures 4E, F**). Thus, we propose that inhibition of NF-κB contributes to the preservation of cardiac function afforded by baricitinib in sepsis.

STAT3 has also been demonstrated to bind the promoter region of NLRP3, thus leading to an increase of NLRP3 protein expression (57) and other experimental findings have convincingly shown that the assembly and activation of the NLRP3 inflammasome is linked to activation of the JAK/STAT pathway (58–61). As widely documented, NLRP3 inflammasome plays a pivotal role in sepsis by driving the formation of IL-1β and IL-18 (62) and, most notably, inhibitors of assembly and activation of NLRP3 reduce the sepsis-driven cardiac dysfunction in sepsis (63–66). We report here that inhibition of the activation of the JAK2/STAT3 pathway with baricitinib reduces the activation of NLRP3 inflammasome and the cleavage of pro-caspase-1 in caspase-1 in septic hearts (**Figures 4C, D**). Together, these observations suggest that inhibition of assembly of the NLRP3 inflammasome and release of the cardio-suppressive mediators IL-1β and IL-18 (67) contributes to the preservation of cardiac function afforded by baricitinib in sepsis.

The article "Baricitinib protects mice from sepsis-induced cardiac dysfunction and multiple-organ failure" was retracted in 2024. Reasons: duplicated images; unreliable data; unreliable results or conclusions; concerns about the images.

In addition to the efficacy of baricitinib and mechanism of action of this JAK1/JAK2-inhibitor in sepsis, we also evaluated any potential gender differences in either degree of cardiac and organ dysfunction/injury, or treatment response. We report here for the first time that the degree of protection afforded by baricitinib is similar in both male and female mice with sepsis (**Figures 5A–D**). In particular, the degree of activation of the JAK2/STAT3 pathway by sepsis in the heart and the degree of preservation of cardiac function afforded by baricitinib were similar in both genders (**Figures 4A, B**). Similarly, the degree of activation of the NLRP3 inflammasome and NF-κB pathways in the heart were qualitatively similar in male and female mice with sepsis, as was the inhibition by baricitinib of these pathways (**Figures 4C–F**). These results reflect what we obtained by the statistical analysis of the clinical data from septic shock patients (**Figures 1C, D**).

## Limitations of the study

This study does not investigate the effects of baricitinib on the mortality caused by sepsis, which is the FDA-approved primary efficacy endpoint for clinical trials in patients with sepsis. Unfortunately, our UK HO license does not permit us to use mortality as primary endpoint of our sepsis efficacy studies. In our study, we have, therefore, determined organ dysfunction, MSS and hypothermia as surrogate markers of outcome and, hence, mortality. Although we studied sepsis and drug response in both male and female animals, all animals in this study were young. In mice, the severity of sepsis and organ dysfunction increases both with age and comorbidities including diabetes or chronic kidney disease (55, 68–72). Although sepsis is a key driver of mortality in neonates (73–75), surgical sepsis is more common and more severe in older patients (76, 77) and, hence, further studies in older animals (or larger animals) are warranted.

Moreover, we reported here that the therapeutic effects of baricitinib on sepsis-induced cardiac dysfunction are, at least in part, related to the reduction in the activation of NLRP3 inflammasome and NF-κB pathways in the heart. However, it would be useful to measure the level of pro-inflammatory cytokines systemically to get a better understanding of the ability of the drug to reduce the sepsis-related cytokines storm.

The article "Baricitinib protects mice from sepsis-induced cardiac dysfunction and multiple-organ failure" was retracted in 2024. Reasons: duplicated images; unreliable data; unreliable results or conclusions; concerns about the images.

## Conclusion

In conclusion, all our findings support the view that a) the expression of JAK2 and STAT3 is enhanced in post-operative patients with sepsis, and b) activation of the JAK2/STAT3 pathway plays a crucial role in the pathophysiology of sepsis-induced cardiac dysfunction and multiple-organ failure in both male and female mice. As there is recent clinical evidence that baricitinib has beneficial effects in patients with COVID-19 (viral sepsis), we propose that this FDA-approved drug may be of benefit in patients with trauma (33), trauma-associated sepsis (this study) and indeed bacterial sepsis.

## Data availability statement

The raw data supporting the conclusions of this article will be made available by the authors, without undue reservation.

## Ethics statement

Ethical approval was not required for the study involving humans in accordance with the local legislation and institutional requirements. Written informed consent to participate in this study was not required from the participants or the participants’ legal guardians/next of kin in accordance with the national legislation and the institutional requirements. The animal study was approved by The Animal Welfare Ethics Review Board of Queen Mary University of London (QMUL) approved all the *in vivo* experiments in accordance with the Home Office guidance on the Operation of Animals (Scientific Procedures Act 1986) published by Her Majesty’s Stationery Office and the Guide for the Care and Use of Laboratory Animals of the National Research Council. All research was conducted under U.K. Home Office project license number PP6747232. All *in vivo* experiments are reported in accordance to ARRIVE guidelines. The study was conducted in accordance with the local legislation and institutional requirements.

## Author contributions

Concept and design: CV, CT and SM. Acquisition, analysis, or interpretation of data: CV, SM, GA, EP, SC, MC, and CT. Drafting the manuscript: CV and CT. All authors contributed to the article and approved the submitted version.
